The article "Modelling the COVID-19 Mortality Rate with a New Versatile Modification of the Log-Logistic Distribution" was published in 2021. Journal: Comput Intell Neurosci.

# Modelling the COVID-19 Mortality Rate with a New Versatile Modification of the Log-Logistic Distribution

**DOI:** 10.1155/2021/8640794

**Published:** 2021-11-13

**Authors:** Abdisalam Hassan Muse, Ahlam H. Tolba, Eman Fayad, Ola A. Abu Ali, M. Nagy, M. Yusuf

**Affiliations:** ^1^Department of Mathematics (Statistics Option) Programme, Pan African University, Institute of Basic Science, Technology and Innovation (PAUSTI), Nairobi 6200-00200, Kenya; ^2^Department of Mathematics, Faculty of Science, Mansoura University, Mansoura 35516, Egypt; ^3^Department of Biotechnology, College of Science, Taif University, P.O. Box 11099, Taif 21944, Saudi Arabia; ^4^Department of Chemistry, College of Science, Taif University, P.O. Box 11099, Taif 21944, Saudi Arabia; ^5^Department of Statistics and Operation Research, Faculty of Science, King Saud University, Riyadh, Saudi Arabia; ^6^Department of Mathematics, Faculty of Science, Fayoum University, Fayoum, Egypt; ^7^Department of Mathematics, Faculty of Science, Helwan University, Cairo, Egypt

## Abstract

The goal of this paper is to develop an optimal statistical model to analyze COVID-19 data in order to model and analyze the COVID-19 mortality rates in Somalia. Combining the log-logistic distribution and the tangent function yields the flexible extension log-logistic tangent (LLT) distribution, a new two-parameter distribution. This new distribution has a number of excellent statistical and mathematical properties, including a simple failure rate function, reliability function, and cumulative distribution function. Maximum likelihood estimation (MLE) is used to estimate the unknown parameters of the proposed distribution. A numerical and visual result of the Monte Carlo simulation is obtained to evaluate the use of the MLE method. In addition, the LLT model is compared to the well-known two-parameter, three-parameter, and four-parameter competitors. Gompertz, log-logistic, kappa, exponentiated log-logistic, Marshall–Olkin log-logistic, Kumaraswamy log-logistic, and beta log-logistic are among the competing models. Different goodness-of-fit measures are used to determine whether the LLT distribution is more useful than the competing models in COVID-19 data of mortality rate analysis.

## 1. Introduction

Models are at the heart of almost all statistical work. A statistical model is a classification of probability distributions. The distribution family can be parametric, semiparametric, or nonparametric. Parametric models produce more efficient estimates with lower standard errors than nonparametric and semiparametric models [1], more specifically, if the distributional assumption is correct. In general, probability distributions have been widely used to model lifetime data in a variety of fields, particularly biomedical sciences and engineering. Because of the variability of the data, the statistical models chosen have a significant impact on the quality of the modelling in terms of providing the best description of the phenomenon under consideration.

The generated family of distributions has a large influence on the quality of statistical analysis procedures, and much effort has gone into developing new statistical models. There are, however, a number of significant issues with actual data that do not fit into any of the commonly used mathematical models. As a result, the technique of extending a family of distributions by introducing new parameters is acknowledged in the statistical literature.

The log-logistic distribution is an excellent choice for analyzing data with unimodal or decreasing failure rates. However, in a number of situations where data behave monotonically, such as increasing failure rates, or nonmonotonically, such as bathtub- or modified bathtub-shaped failure rates, the log-logistic model is not a good candidate model to use [2–5]. As a result, new extensions and generalizations to existing models are required for accurate and precise data modelling. As a result, numerous statistical techniques are intended to discover new modifications to classical models in order to achieve a better fit to the data of interest. Other techniques, on the other hand, such as the Sin-G family, Cos-G family, Tan-G family, and Sec-G family, provide a versatile generalization of the existing probability distribution without adding any extra parameters [6–10]. The techniques that are effectively used to extend the classical distributions without adding extra parameters are termed as “new trigonometric classes of probability distribution” [11].

A random variable *X* is said to have a log-logistic distribution with shape parameter *β* > 0 and scale parameter *α* > 0,  denoted by *X* ∼ LLog (*α*,  *β*), if its cumulative distribution function (cdf) is defined by the following equation:

(1) $$\begin{array}{c} F\left(x;\varphi \right)=\;\frac{{\left(x/\alpha \right)}^{\beta }}{1+{\left(x/\alpha \right)}^{\beta }},\;x\geq 0,\;\varphi >0. \end{array}$$

The probability density function (pdf) is given by

(2) $$\begin{array}{c} f\left(x;\;\varphi \right)=\;\frac{\left(\beta /\alpha \right){\left(x/\alpha \right)}^{\beta -1}}{{\left(1+{\left(x/\alpha \right)}^{\beta }\right)}^{2}},\;x\geq 0,\;\varphi >0. \end{array}$$

The reliability (survival) function is given by

(3) $$\begin{array}{c} S\left(x;\;\varphi \right)=1-F\left(x;\;\varphi \right)=\;\frac{{\left(x/\alpha \right)}^{-\beta }}{1+{\left(x/\alpha \right)}^{-\beta }},\;x\geq 0,\;\varphi >0. \end{array}$$

The failure (hazard) rate function is given by

(4) $$\begin{array}{c} h\left(x;\varphi \right)=\frac{f\left(x;\varphi \right)}{S\left(x;\varphi \right)}=\;\frac{f\left(x;\varphi \right)}{1-F\left(x;\varphi \right)}\;=\;\frac{\left(\beta /\alpha \right){\left(x/\alpha \right)}^{\beta -1}}{1+{\left(x/\alpha \right)}^{\beta }},\;\;x\geq 0,\;\varphi >0. \end{array}$$

The reversed hazard rate function (also known as the retro function) is given by

(5) $$\begin{array}{c} r\left(x;\;\varphi \right)=\frac{f\left(x;\;\varphi \right)}{F\left(x;\;\varphi \right)}\frac{\left[\left(\beta /\alpha \right){\left(x/\alpha \right)}^{\beta -1}/{\left(1+{\left(x/\alpha \right)}^{\beta }\right)}^{2}\right]}{\left[{\left(x/\alpha \right)}^{\beta }/\left(1+{\left(x/\alpha \right)}^{\beta }\right)\;\right]}\;=\frac{\left(\theta /\alpha \right){\left(x/\alpha \right)}^{-1}}{1+{\left(x/\alpha \right)}^{\beta }};\;\;x\geq 0,\;\varphi >0. \end{array}$$

The cumulative hazard rate function is given by

(6) $$\begin{array}{c} H\left(x\right)=\;-\log\;S\left(x;\phi \right)=-\log\left(\frac{{\left(x/\alpha \right)}^{-\beta }}{1+{\left(x/\alpha \right)}^{-\beta }}\;\right),\;x\geq 0,\;\phi >0, \end{array}$$

where *ϕ*=(*α*, *β*)′ is a vector of parameters.

It is well understood that the classical log-logistic distribution fails to capture the accurate phenomenon under investigation in many cases. As a result, several modifications have been proposed and researched. Inducting one or more parameters to the classical log-logistic distribution yields a modified form of the log-logistic distribution. When compared to the classic log-logistic distribution, several of these modified distributions have been found to be more flexible and adaptable of modelling real-life data. An up-to-date survey of recent modifications of the log-logistic distribution can be found in [12].

Most modifications of the log-logistic model in the statistical literature have been derived by adding extra parameters to control the shape of the skewness (or asymmetry) and the kurtosis of the distribution; see the exponentiated LL distribution [13], beta LL distribution [14], gamma LL distribution [15], Marshall–Olkin LL distribution [16], transmuted LL distribution [17], cubic transmuted LL distribution [18], McDonald LL distribution [19], and alpha power transformed LL distribution [20, 21]. Other generalizations and modifications of the log-logistic distribution developed recently can be seen in [22, 23].

The majority of techniques for extending the classical LL model produce a heavy-tailed distribution. Unfortunately, the abovementioned generalizations of the log-logistic distribution have some limitations. For instance, (i) adding extra parameter(s) to the distribution enhances flexibility, but even so, such practices usually result in reparameterization issues; (ii) the number of model parameters is increased, causing difficulty in estimating the model's parameters; (iii) some extending techniques reduce the tractability of the cdf, making manual computation of statistical properties more difficult; and (iv) other generalization techniques complicate the pdf, resulting in computational issues; incorporating new extra parameters into existing models increases flexibility, which is a desirable feature. On the other hand, it makes inferences more difficult [24, 25]. As a result, in this study, we modified the classical log-logistic distribution with a two-parameter continuous distribution referred to the log-logistic tangent distribution (LLT).

The primary goal of this current study is it to introduce and investigate a versatile modification of the log-logistic distribution using the Tan-G family generator method. As previously stated, the proposed two-parameter distribution may be more flexible than other popular log-logistic model extensions. It would eventually become clear that the proposed distribution family accommodates both monotone and nonmonotone hazard rates.

The rest of the paper is organized as follows. The proposed family is discussed in Section 2.  Section 3 presents the proposed distribution. Some mathematical and statistical properties of the proposed distribution are discussed in Section 4.  Section 5 presents the estimation of the unknown parameters of the model.  Section 6 discusses a Monte Carlo simulation for the proposed model. In Section 7, an application to a real-life dataset is presented and discussed. The comparison of some of the parametric probability distributions and their submodels is presented. Finally, concluding remarks and a work summary are presented in Section 8.

## 2. The Proposed Family

Several continuous probability distributions involving trigonometric functions have been developed in the statistics literature by many researchers, with the tangent distribution being notable due to its wide range of applications in many real-life datasets from various disciplines. A useful survey in this context can be found in [11, 24–27]. In this study, we concentrate on the trigonometric classes of continuous probability distributions, which are described by a cdf concerning trigonometric functions (tangent, cosine, sine, secant, and different mixtures of them). The Tan-G family developed in [11, 26–29] is the fundamental work.

As indicated by its name, Souza et al. [28] introduced a new method for extending the classical probability distributions, leading to greater flexibility in analyzing and modelling different data types. They looked at a parent distribution, which is an arbitrary continuous probability distribution with a cdf and a corresponding pdf. The cumulative distribution function (cdf) is defined by the associated tangent family of distributions.

(7) $$\begin{array}{c} F_{\text{Tan}}\left(x\right)=\;\int_{0}^{\pi /4G\left(x\right)}\sec^{2}\left(t\right)dt. \end{array}$$

Equation (7) can be written as

(8) $$\begin{array}{c} F_{\text{Tan}}\left(x\right)=\tan\left(\frac{\pi }{4}\;G\left(x\right)\right), \end{array}$$

where *G*(*x*) is the cdf of the parent (baseline) distribution, and if *G*(*x*) has pdf *g*(*x*), the pdf of the class is given by

(9) $$\begin{array}{c} f_{\text{Tan}}\left(x\right)=\frac{\pi }{4}\;g\left(x\right)\;\sec^{2}\left(\frac{\pi }{4}\;G\left(x\right)\right). \end{array}$$

The survival function is obtained by

(10) $$\begin{array}{c} S_{\text{Tan}}\left(x\right)=1-\;\tan\left(\frac{\pi }{4}\;G\left(x\right)\right). \end{array}$$

The failure rate function is given by

(11) $$\begin{array}{c} h_{\text{Tan}}\left(x\right)=\frac{f_{\text{Tan}}\left(x\right)}{S_{\text{Tan}}\left(x\right)}=\;\frac{\pi /4\;g\left(x\right)\sec^{2}\left(\pi /4G\left(x\right)\right)\;}{1-\tan\left(\pi /4\;G\left(x\right)\right)}. \end{array}$$

The reversed hazard rate function is given by

(12) $$\begin{array}{c} r_{\text{Tan}}\left(x\right)=\frac{f_{\text{Tan}}\left(x\right)}{F_{\text{Tan}}\left(x\right)}=\;\frac{\pi /4g\left(x\right)\sec^{2}\left(\pi /4G\left(x\right)\right)\;}{\tan\left(\pi /4\;G\left(x\right)\right)}. \end{array}$$

Also, the cumulative hazard rate function is given by

(13) $$\begin{array}{c} H_{\text{Tan}}\left(x\right)=-\log\;S_{\text{Tan}}\left(x\right)=\;-\log\left\{1-\;\tan\left(\frac{\pi }{4}\;G\left(x\right)\right)\right\}. \end{array}$$

Recently, Souza et al. [28] proposed and studied the Burr-XII tangent distribution which serves as a potential lifetime model. Ampadu [29] introduced and studied the Weibull tangent distribution with applications to health science data. Hence, the Tan-G family is a special family for extending the classical well-known lifetime distributions without adding an extra parameter.

## 3. The Log-Logistic Tangent Distribution

In this section, the LLT distribution has been examined, considering that *G*(*x*) is the cdf of the log-logistic distribution.

The distribution function (cdf) of the log-logistic tangent distribution, for *x* > 0,   can be expressed as

(14) $$\begin{array}{c} F_{\text{Tan}-LL}\left(x;\;\phi \right)=\tan\left\{\frac{\pi }{4}\;\left(\frac{{\left(x/\alpha \right)}^{\beta }}{1+{\left(x/\alpha \right)}^{\beta }}\right)\right\}. \end{array}$$

The corresponding probability density function to the abovementioned cdf is given by

(15) $$\begin{array}{c} f_{\text{Tan}-LL}\left(x;\;\phi \right)=\frac{\pi }{4}\;\left\{\frac{\left(\beta /\alpha \right){\left(x/\alpha \right)}^{\beta -1}}{{\left(1+{\left(x/\alpha \right)}^{\beta }\right)}^{2}}\right\}\;\sec^{2}\left\{\frac{\pi }{4}\;\left(\frac{{\left(x/\alpha \right)}^{\beta }}{1+{\left(x/\alpha \right)}^{\beta }}\right)\right\}. \end{array}$$

The survival function is expressed as follows:

(16) $$\begin{array}{c} S_{\text{Tan}-LL}\left(x;\;\phi \right)=1-\;\tan\left\{\frac{\pi }{4}\;\left(\frac{{\left(x/\alpha \right)}^{\beta }}{1+{\left(x/\alpha \right)}^{\beta }}\right)\right\}. \end{array}$$

The hazard rate function is obtained by

(17) $$\begin{array}{c} h_{\text{Tan}-LL}\left(x;\;\phi \right)=\frac{\pi /4\;\left\{\left(\beta /\alpha \right){\left(x/\alpha \right)}^{\beta -1}/{\left(1+{\left(x/\alpha \right)}^{\beta }\right)}^{2}\right\}\;\sec^{2}\left\{\pi /4\;\left({\left(x/\alpha \right)}^{\beta }/1+{\left(x/\alpha \right)}^{\beta }\right)\right\}}{1-\tan\left\{\pi /4\;\left({\left(x/\alpha \right)}^{\beta }/1+{\left(x/\alpha \right)}^{\beta }\right)\right\}}. \end{array}$$

The reversed hazard rate function is expressed as follows:

(18) $$\begin{array}{c} r_{\text{Tan}-LL}\left(x;\;\phi \right)=\frac{\pi /4\;\left\{\left(\beta /\alpha \right){\left(x/\alpha \right)}^{\beta -1}/{\left(1+{\left(x/\alpha \right)}^{\beta }\right)}^{2}\right\}\;\sec^{2}\left\{\pi /4\;\left({\left(x/\alpha \right)}^{\beta }/1+{\left(x/\alpha \right)}^{\beta }\right)\right\}}{\tan\left\{\pi /4\;\left({\left(x/\alpha \right)}^{\beta }/1+{\left(x/\alpha \right)}^{\beta }\right)\right\}}. \end{array}$$

The cumulative hazard function can be given as follows:

(19) $$\begin{array}{c} H_{\text{Tan}-LL}\left(x\right)=-\log\;S_{\text{Tan}-LL}\left(x\right)=\;-\log\left[1-\;\tan\left\{\frac{\pi }{4}\;\left(\frac{{\left(x/\alpha \right)}^{\beta }}{1+{\left(x/\alpha \right)}^{\beta }}\right)\right\}\right]. \end{array}$$

With *x* ≥ 0,  *α*, *β* > 0, and*φ*=(*α*, *β*)′ is the vector parameter in all of the abovementioned equations, respectively.

Some possible shapes of the pdf, cdf, hazard function, survival function, and the reversed hazard functions of the log-logistic tangent distribution are displayed in Figures 1–7.

The hazard rate function of the proposed distribution can accommodate for both monotone (increasing and decreasing) and nonmonotone (i.e., unimodal) hazard rates, as it can be seen in Figures 4–6, and Figure 7 represents the reversed hazard function of the LLT distribution.

## 4. Some Statistical Properties of the Proposed Distribution

In this section, we use numerical examples to derive some mathematical properties of the log-logistic tangent distribution, such as the quantile function, skewness and kurtosis, moments, and residual and reverse residual life.

### 4.1. Quantile Function

For this model, the quantile function of the LLT distribution is used in theoretical aspects of distribution theory such as statistical simulations and applications. To generate random samples, the simulation algorithm used a quantile function by following the steps in Algorithm 1.

Let *X* be the Tan-G-distributed random variable. The quantiles can be utilized to obtain data of the distribution according to

(20) $$\begin{array}{c} x=Q\left(u\right)=\;F^{-1}\left(u\right)=\;G^{-1}\left[\frac{4}{\pi }\arctan\left(u\right)\right]. \end{array}$$

The LLT distribution's quantile function is given by

(21) $$\begin{array}{c} Q_{\text{LLT}}\left(u\right)=\;\alpha {\left(\frac{4/\pi \arctan\left(u\right)}{1-4/\pi \arctan\left(u\right)}\right)}^{\frac{1}{\beta }}. \end{array}$$

The lower quartile (*Q*1), median (*Q*2), and upper quartile (*Q*3) of LLT distribution can be derived from the equation of the quantile function by setting *u*=1/4, 1/2,  and 3/4, respectively.

The quantiles of the LLT distribution for some parameter values are shown in Table 1.

### 4.2. Skewness and Kurtosis

Some of the properties of the continuous distribution can be studied through its asymmetry and kurtosis. The mathematical form of the Moors Kurtosis and Galton asymmetry (or skewness) of the LLT model with two parameters is defined by the following relationship:

(22) $$\begin{array}{c} S_{K}=\;\frac{Q\left(3/4\right)\;+Q\left(1/4\right)\;-2Q\left(2/4\right)}{Q\left(3/4\right)-Q\left(1/4\right)},\;\\ K_{M}=\;\frac{Q\left(7/8\right)\;+Q\left(3/8\right)\;-Q\left(5/8\right)-Q\left(1/8\right)}{Q\left(6/8\right)-Q\left(2/8\right)}, \end{array}$$

where *Q* describes different quartile values.

The equations above can be solved as functions of the LLT quantile function. These measures have the advantage of being less sensitive in the presence of outliers and existing even when the distribution is devoid of moments.

### 4.3. Moments

Moments are essential in statistical modelling, particularly in role in applications. The LLT distribution's *r*th moment is defined as

(23) $$\begin{array}{c} \mu_{r}^{\prime }=\;\int_{-\infty }^{\infty }x^{r}f\left(x;\alpha ,\beta \right)dx. \end{array}$$

In fact, we have

(24) $$\begin{array}{c} \mu_{r}^{\prime }=\;\int_{-\infty }^{\infty }x^{r}\frac{\pi }{4}\;\left\{\frac{\left(\beta /\alpha \right){\left(x/\alpha \right)}^{\beta -1}}{{\left(1+{\left(x/\alpha \right)}^{\beta }\right)}^{2}}\right\}\;\sec^{2}\left\{\frac{\pi }{4}\;\left(\frac{{\left(x/\alpha \right)}^{\beta }}{1+{\left(x/\alpha \right)}^{\beta }}\right)\right\}dx. \end{array}$$

The first five moments followed by the standard deviation, coefficient of variance, skewness, and kurtosis for some parameter values are shown in Table 2.

### 4.4. Residual Life and Reverse Residual Life

The residual lifetime function (rlf) has broader uses in risk management and survival analysis. The rlf of the LLT random variable (r.v.) can be expressed as follows:

(25) $$\begin{array}{c} R_{\left(t\right)\;}\left(x\right)=\;\frac{S\left(x+t\right)}{S\left(t\right)},\\ R_{\left(t\right)\;}\left(x\right)=\frac{1-\tan\left\{\pi /4\;\left({\left(x+t/\alpha \right)}^{\beta }/\left(1+{\left(\left(x+t\right)/\alpha \right)}^{\beta }\right)\right)\right\}}{1-\tan\left\{\pi /4\;\left({\left(x/\alpha \right)}^{\beta }/\left(1+{\left(x/\alpha \right)}^{\beta }\right)\right)\right\}\;}. \end{array}$$

Furthermore, the reverse residual lifetime function (rrlf) of the LLT r.v. can be obtained as follows:

(26) $$\begin{array}{c} {\hat{R}}_{\left(t\right)\;}\left(x\right)=\frac{S\left(x+t\right)}{S\left(t\right)},\;\\ {\hat{R}}_{\left(t\right)\;}\left(x\right)=\frac{1-\tan\left\{\pi /4\;\left({\left(x-t/\alpha \right)}^{\beta }/\left(1+{\left(\left(x-t\right)/\alpha \right)}^{\beta }\right)\right)\right\}}{1-\tan\left\{\pi /4\;\left({\left(x/\alpha \right)}^{\beta }/\left(1+{\left(x/\alpha \right)}^{\beta }\right)\right)\right\}\;}. \end{array}$$

## 5. Estimation of the Parameters

The maximum likelihood approach is used in this section to estimate the unknown parameters of the log-logistic tangent distribution based on a complete sample. Let *x*={*x*_1_, *x*_2_,…,*x*_*n*_}^*T*^ represent *n* independent random variables drawn from the LLT distribution. The sample's likelihood function is defined as

(27) $$\begin{array}{c} L=\;\prod_{i=1}^{n}f\left(x_{i},\;\alpha ,\beta \right),\\ L\left(x;\;\alpha ,\beta \right)=\;\prod_{i=1}^{n}\frac{\pi }{4}\;\left\{\frac{\left(\beta /\alpha \right){\left(x/\alpha \right)}^{\beta -1}}{{\left(1+{\left(x/\alpha \right)}^{\beta }\right)}^{2}}\right\}\;\sec^{2}\left\{\frac{\pi }{4}\;\left(\frac{{\left(x/\alpha \right)}^{\beta }}{1+{\left(x/\alpha \right)}^{\beta }}\right)\right\}. \end{array}$$

The log-likelihood function can be written as follows:

(28) $$\begin{array}{c} \ell =n\;\log\frac{\pi }{4}+n\;\log\;\beta -n\beta \;\log\;\alpha +\left(\beta -1\right)\sum_{i=1}^{n}\log\left(x_{i}\right)-2\sum_{i=1}^{n}\log\left[1+{\left(\frac{x_{i}}{\alpha }\right)}^{\beta }\right]+2\sum_{i=1}^{n}\log\left[\sec\left\{\frac{\pi }{4}\;\left({\left(\frac{x_{i}}{\alpha }\right)}^{\beta }{\left[1+{\left(\frac{x_{i}}{\alpha }\right)}^{\beta }\right]}^{-1}\right)\right\}\right]. \end{array}$$

By taking the 1^st^ derivatives of the log-likelihood function in equation (28) with respect to *α* and *β* parameters and setting the result to zero, we get

(29) $$\begin{array}{c} \frac{\partial \ell }{\partial \alpha }=-\frac{n\beta }{\alpha }+\frac{2\beta }{\alpha }\sum_{i=1}^{n}{\left(\frac{x_{i}}{\alpha }\right)}^{\beta }{\left[1+{\left(\frac{x_{i}}{\alpha }\right)}^{\beta }\right]}^{-1}\;-\;\frac{\pi }{2}\;\overset{n}{\underset{i=1}{\sum }}{\left(\frac{x_{i}}{\alpha }\right)}^{\beta }\left(\frac{\beta }{\alpha }\right){\left[1+{\left(\frac{x_{i}}{\alpha }\right)}^{\beta }\right]}^{-2}\tan\left\{\frac{\pi }{4}\;\left({\left(\frac{x_{i}}{\alpha }\right)}^{\beta }{\left[1+{\left(\frac{x_{i}}{\alpha }\right)}^{\beta }\right]}^{-1}\right)\right\},\\ \frac{\partial \ell }{\partial \beta }=\frac{n}{\beta }-n\;\log\left(\alpha \right)+\;\sum_{i=1}^{n}\log\left(x_{i}\right)-2\sum_{i=1}^{n}{\left(\frac{x_{i}}{\alpha }\right)}^{\beta }\log\left(\frac{x_{i}}{\alpha }\right){\left[1+{\left(\frac{x_{i}}{\alpha }\right)}^{\beta }\right]}^{-1}+\;\frac{\pi }{2}\;\sum_{i=1}^{n}{\left(\frac{x_{i}}{\alpha }\right)}^{\beta }\log\left(\frac{x_{i}}{\alpha }\right)\;\left(\frac{x_{i}}{\alpha }\right){\left[1+{\left(\frac{x_{i}}{\alpha }\right)}^{\beta }\right]}^{-2}\;\tan\left\{\frac{\pi }{4}\;\left({\left(\frac{x_{i}}{\alpha }\right)}^{\beta }{\left[1+{\left(\frac{x_{i}}{\alpha }\right)}^{\beta }\right]}^{-1}\right)\right\}\;. \end{array}$$

It is worth noting that the MLE's $\hat{\alpha }\text{ and }\hat{\beta }$ of *α* and *β*,  respectively, can be achieved by equating the outcomes to zero and solving the system of nonlinear equations numerically. The well-known theory on MLE can be used under some standard regularity conditions, ensuring nice asymptotic properties [30].

## 6. Simulation Study

In this section, we use Monte Carlo (MC) simulation to evaluate the effectiveness of the Maximum Likelihood Estimation (MLE) method for estimating the log-logistic tangent distribution parameters. The simulation study is carried out to investigate the average bias (AB), mean square error (MSE), and root mean square error (RMSE) for the parameters of the proposed model. The simulation experiment was conducted by running a number of simulations with varying sample sizes and parameter values. The quantile function given in Eq. (21) was used to generate random samples for the LLT. The MC simulation study was iterated 750 times with sample sizes *n*=25,  50,   …, 750 and the parameter scenarios *α*=2.0  and *β*=1.5 in set I and *α*=3.0  and *β*=2.0 in set II.

The MLEs are ascertained for each item of simulated data, say ($\hat{\alpha },\hat{\beta }$) for *i*=1,2,…,  750, and the AB, MSEs, and RMSEs of the parameters were calculated by

(30) $$\begin{array}{c} \text{AB}=\;\frac{1}{N}\sum_{i=1}^{N}\left(\hat{\theta }-\theta \right),\;\\ \text{MSE}=\;\frac{1}{N}\sum_{i=1}^{N}{\left(\hat{\theta }-\theta \right)}^{2},\\ \text{RMSE}=\;\sqrt{\frac{1}{N}\sum_{i=1}^{N}{\left(\hat{\theta }-\theta \right)}^{2}},\; \end{array}$$

where *θ*=*α* and *β*.

Table 3 shows the AB, MSE, and RMSE values of the parameters for various sample sizes. Based on these results, we draw the conclusion that MLEs do a good job of estimating parameters and that the estimates seem to be reasonably constant and closer to the true values for these sample sizes. In addition, Table 4 shows that the RMSE decreases as the sample size increases, as expected. Furthermore, as sample size increases, so does the AB. As a result, even if the sample size is small, the MLEs and their asymptotic results can be used to calculate confidence intervals for model parameters.

The simulation results for the aforementioned measures are depicted in Figures 8 and 9. These plots demonstrate that increasing the sample size *n* reduces the estimated biases. Furthermore, as the sample size *n* is increased, the estimated MSEs and RMSEs decay toward zero. These findings demonstrate the MLEs' efficiency as well as their consistency.

## 7. Applications to the COVID-19 Dataset

The log-logistic tangent distribution derivation's main interest is its application in data analysis goals, which makes it valuable in different disciplines, especially those associated with mortality data analysis. A number of proposed distributions for COVID-19 datasets have recently been proposed; for more information on these, please see [31–39].

The log-logistic tangent distribution was applied to a real-life COVID-19 mortality rate dataset from Somalia for demonstration purposes, and its performance was compared to the performance of other fitted models such as the log-logistic, Weibull, Gompertz, and kappa distributions. For the log-likelihood, the most common information criteria including Akaike Information Criterion (AIC), Hannan–Quinn Information Criterion (HQIC), Corrected Akaike Information Criterion (CAIC), and Bayesian Information Criterion (BIC) values were used to select the most appropriate. The Anderson–Darling (*A*^∗^) statistic, the Cramer–von Mises (*W*^∗^) distance value, and the Kolmogorov–Smirnov (*K*–*S*) statistic, as well as the corresponding *p* value, are all recorded.

(1) Log-logistic:
  (31) $$\begin{array}{c} f\left(x\right)=\;\frac{\beta /\alpha {\left(x/\alpha \right)}^{\beta -1}}{{\left[1+{\left(x/\alpha \right)}^{\beta }\right]}^{2}},\;\text{ for }x\geq 0. \end{array}$$
(2) Gompertz distribution:
  (32) $$\begin{array}{c} f\left(x\right)=\alpha \beta \;\exp\left(\beta +\alpha x-\beta e^{\alpha x}\right),\;\text{ for }x\geq 0. \end{array}$$
(3) Kappa distribution:
  (33) $$\begin{array}{c} f\left(x\right)=\;\frac{\alpha }{\beta }{\left[\alpha +{\left(\frac{x}{\beta }\right)}^{\alpha }\right]}^{-\left(\alpha +1\right)/\alpha },\;\text{ for }x\geq 0. \end{array}$$

See also the other four recently modified log-logistic distributions with three parameters and four parameters [14, 16, 40, 41].

The AIC is

(34) $$\begin{array}{c} \text{ AIC}=2k-2l. \end{array}$$

The BIC is

(35) $$\begin{array}{c} \text{ BIC}=kln\left(n\right)-2l. \end{array}$$

The CAIC is

(36) $$\begin{array}{c} \text{CAIC}=\frac{2nk}{n-k-1}-2l. \end{array}$$

The HQIC is

(37) $$\begin{array}{c} \text{HQIC}=2kln\left(\ln\left(n\right)\right)-2l, \end{array}$$

where the log-likelihood function is represented by *l*, the sample size by *n*, and the number of model parameters by *k*. The following goodness-of-fit measures are being considered.

The Anderson–Darling (*A*∗) test statistic is given by

(38) $$\begin{array}{c} A^{*}=-n-\frac{1}{n}\sum_{i=1}^{n}\left(2l-1\right)\times \left[\ln\;G\left(X_{i}\right)+\ln\left\{1-G\left(X_{n-i+1}\right)\right\}\right]. \end{array}$$

The Cramer–von Mises (*W*∗) test statistics is given by

(39) $$\begin{array}{c} W^{*}=\frac{1}{12n}+\sum_{i=1}^{n}{\left[\frac{2i-1}{2n}+G\left(X_{i}\right)\right]}^{2}, \end{array}$$

where *x*_*i*_ is the *i*th observation in the sample and *n* is the sample size. When the data are sorted in ascending order, *x*_*i*_ is calculated.

The best model has the lowest AIC, CAIC, BIC, and HQIC, a well as the lowest *A*∗, *W*∗, and *K*–*S* values. In addition, the best model is chosen as the one with the highest log-likelihood function value, and *p* values for the *K*–*S* statistics are applied to compare the competitive distributions.

### 7.1. Data I : Somalia COVID-19 Mortality Rate Dataset

The dataset contains COVID-19 mortality rate from Somalia during the time between 1^st^ March 2021 to 20^th^ April 2021 (see https://covid19.who.int/). These data are made up of a rough mortality rate. The data frame contains 51 observations, which are formed by using the daily cumulative cases (DCCs) and daily new deaths (DNDs). The data are as follows:

3.008, 2.963, 4.762, 5.263, 11.382, 5.330, 10.471, 2.857, 4.274, 8.633, 5.882, 10.280, 5.330, 8.730, 7.377, 8.696, 8.257, 4.294, 5.330, 6.769, 11.627, 8.547, 9.302, 7.742, 6.173, 6.015, 5.330, 9.770, 5.330, 4.294, 5.330, 8.120, 7.547, 7.563, 5.330, 6.875, 8.800, 11.429, 5.330, 9.898, 5.330, 5.330, 9.630, 3.750, 5.330, 11.808, 5.330, 5.330, 5.330, 5.785, and 3.265.

### 7.2. Exploratory Data Analysis

The primary goal of data analysis is to extract information from the data. We used five different techniques to perform exploratory data analysis in this work: (1) data descriptive statistics; (2) Box plot; (3) TTT plot; (4) histogram; and (5) time-series plot.  Figure 10 displays the Box, TTT, histogram, and times-series plots for our dataset.

The total-time-on-test (TTT) plot is a graphical method for determining the failure rate function's shape. There is qualitative information about the shape of the failure rate function in many real-world applications that can aid in the selection of a particular distribution. The TTT plot for our dataset in this work is shown, and it shows an increasing failure rate shape.

Table 4 shows us the descriptive statistics of the COVID-19 data for mortality rate between 1^st^ March to 20 April 2021 by computing specific aspects of the data (central tendency and spread).

The proposed LLT distribution has the lowest AIC, CAIC, BIC, and HQIC values and the highest log-likelihood values in Table 5, so it is selected as the most suitable model among the competing distributions considered in this work.

Table 6 shows the parameter estimate and *p* value for the Cramer–von Mises (W∗), Anderson–Darling (A∗), and Kolmogorov–Smirnov (K–S) tests for all competing distributions using abovementioned dataset I. According to Table 6, the proposed LLT distribution has the lowest A∗, W∗, and K–S tests, as well as the highest *p* value. As a result, among the competing distributions considered in this study, the proposed LLT distribution is chosen as the most appropriate model.

The estimated pdf for the competing models is shown in Figure 11, the estimated cdf for the competing models is shown in Figure 12, and the estimated cdf, Kaplan–Meier, pdf, and PP plots for the proposed model are shown in Figure 13.

## 8. Conclusions

The two-parameter log-logistic model has found widespread use in statistical sciences, especially survival analysis, biomedical sciences, engineering, and actuarial sciences. In this paper, we proposed a new probability distribution that derives from a combination of log-logistic distribution and a Tan-G trigonometric class of distribution. This model was named log-logistic tangent distribution “LLT distribution” and has been successfully extended in this work. Reliability function, pdf, cdf, failure rate function, reversed failure rate function, and the cumulative failure rate function were carefully derived, and expressions for the basic statistical properties for the log-logistic tangent distribution have been developed. The log-logistic tangent distribution was applied to the COVID-19 mortality rate dataset and provided a better fit than the known two-parameter, three-parameter, and four-parameter competitors. Gompertz, log-logistic, kappa, exponentiated log-logistic, Marshall–Olkin log-logistic, Kumaraswamy log-logistic, and beta log-logistic based on goodness-of-fit tests, selection criteria such as AIC, BIC, CAIC, and HQIC values, and the log-likelihood value were applied. We, therefore, conclude that the log-logistic tangent distribution is the most adequate model among the ones considered, as well as a very competitive model for describing different datasets in different areas of application.

## Figures and Tables

**Figure 1:** Visual display plots of the cdf of the LLT distribution.

**Figure 2:** Visual display plots of the pdf of the LLT distribution.

**Figure 3:** Plots of the survival function of the LLT distribution.

**Figure 4:** Unimodal hazard rate of the LLT distribution.

**Figure 5:** Plots of the LLT increasing hazard rate.

**Figure 6:** Plots of the LLT decreasing hazard rate.

**Figure 7:** Plots of the retro hazard function of the LLT distribution.

**Figure 8:** MLEs, MSEs, biases, and RMSE plots of the proposed distribution for set I values.

**Figure 9:** MLEs, MSEs, biases, and RMSE plots of the proposed distribution for set II values.

**Figure 10:** Box plot, TTT plot, histogram, and time-series plot for dataset I.

**Figure 11:** Some fitted pdf's of the fitted distributions in dataset I.

**Figure 12:** Some fitted cdf's of the fitted distributions in dataset I.

**Figure 13:** The estimated cdf, Kaplan–Meier, estimated pdf, and PP plots of the log-logistic tangent distribution for dataset I.

**Algorithm 1:** Random generator for the Tan-G class.

**Table 1:** The quantiles of the LLT distribution for some values of the parameters.

Quantiles	(*α*, *β*)				
	(0.5, 1.5)	(0.2, 0.9)	(0.3, 0.8)	(0.1, 1.2)	(0.05, 0.9)
0.1	0.1382	0.0235	0.0269	0.0201	0.0059
0.2	0.2415	0.0595	0.0767	0.0403	0.0149
0.3	0.3518	0.1113	0.1551	0.0644	0.0278
0.4	0.4797	0.1867	0.2776	0.0950	0.0467
0.5	0.6379	0.3001	0.4737	0.1356	0.0751
0.6	0.8473	0.4818	0.8065	0.1933	0.1204
0.7	1.1518	0.8036	1.4343	0.2838	0.2009
0.8	1.6688	1.4908	2.8745	0.4511	0.3727
0.9	2.8956	3.7351	8.0781	0.8983	0.9338

**Table 2:** First five moments, SD, CV, asymmetry, and kurtosis of the LLT distribution for different parameter values.

Moments	(*α*, *β*)				
	(1.1, 0.)	(1.2, 0.9)	(0.3, 0.8)	(0.1, 1.2)	(0.2, 0.4)
*μ*′_1_	0.1383	0.1445	0.1727	0.1772	0.0920
*μ*′_2_	0.0804	0.0862	0.0914	0.0744	0.0471
*μ*′_3_	0.0562	0.0608	0.0611	0.0440	0.0314
*μ*′_4_	0.0431	0.0469	0.0457	0.0306	0.0236
*μ*′_5_	0.0349	0.0381	0.0364	0.0234	0.0188
*SD*	0.2476	0.2555	0.2482	0.2074	0.1965
*CV*	1.7906	1.7685	1.4377	1.1709	2.1388
*CS*	1.8534	1.7702	1.5728	1.7408	2.6374
CK	5.3540	4.9762	4.5195	5.6950	9.5119

**Table 3:** MC simulation outcomes for the proposed distribution using the values for MLEs, ABs, MSEs, and RMSEs.

Parameters		I				II			
	n	MLE	AB	MSE	RMSE	MLE	AB	MSE	RMSE
*α*	25	2.059	0.059	0.273	0.522	3.060	0.060	0.368	0.607
	50	2.030	0.030	0.117	0.341	3.022	0.022	0.142	0.378
	100	2.010	0.010	0.066	0.256	3.017	0.017	0.086	0.294
	200	2.008	0.008	0.030	0.172	3.013	0.013	0.041	0.202
	400	2.004	0.004	0.015	0.124	3.008	0.008	0.019	0.137
	600	2.003	0.003	0.010	0.100	3.003	0.003	0.012	0.108
	700	2.002	0.002	0.007	0.086	3.002	0.002	0.009	0.098

*β*	25	1.584	0.084	0.079	0.282	2.124	0.124	0.156	0.395
	50	1.541	0.041	0.035	0.187	2.060	0.060	0.065	0.255
	100	1.518	0.018	0.017	0.130	2.023	0.023	0.029	0.173
	200	1.513	0.013	0.008	0.089	2.011	0.011	0.014	0.120
	400	1.505	0.005	0.004	0.062	2.007	0.007	0.007	0.085
	600	1.502	0.002	0.003	0.050	2.004	0.004	0.004	0.068
	700	1.501	0.001	0.002	0.044	2.003	0.003	0.003	0.058

**Table 4:** Descriptive measures of data I.

N	Min.	Median	Mode	Variance	Asymmetry	Kurtosis	Mean	Max.	CV	Geo. mean
51	2.857	5.882	5.5	5.962	0.450	−0.732	6.793	11.81	0.359	6.363

**Table 5:** Likelihood and the information criteria for data I.

Distribution	*ℓ*	AIC	BIC	CAIC	HQIC
LLT	−116.839	236.677	240.541	237.927	238.154
LL	−118.198	238.997	241.860	239.246	239.473
Gompertz	−120.495	244.991	248.854	245.8241	246.467
Kappa	−127.196	258.391	262.255	258.641	259.867
Expo LL	−116.995	239.991	245.786	240.501	242.205
Beta LL	−115.559	239.119	246.846	239.988	242.071
Kumw LL	−115.970	239.940	247.667	240.810	242.892
Mo-LL	−116.998	239.996	245.792	240.507	242.212

**Table 6:** MLE model parameter estimators and goodness-of-fit tests for the COVID-19 data.

Distributions	Estimates	*W* ^∗^	*A* ^∗^	**K** − S (*P* value)
LLT (*δ*, *θ*)	*δ* = 5.904 *θ* = 4.814	0.199	1.067	0.169 (0.206)

llog (*α*, *β*)	*α* = 6.388 *β* = 4.633	0.203	1.089	0.169 (0.109)

Gompertz (*α*, *β*)	*α* = 0.365 *β* = 0.021	0.221	1.266	0.181 (0.016)

Kappa (*α*, *β*)	*α* = 58.227 *β* = 11.071	0.322	1.856	0.267 (0.002)

Exp LL (*α*, *β*, *γ*)	*α* = 1.050 *β* = 4.561 *γ* = 6.285	0.210	1.085	0.197 (0.113)

Beta LL (*α*, *β*, *γ*, *δ*)	*α* = 5.431 *β* = 20.368 *γ* = 1.360 *δ* = 17.705	0.214	1.075	0.178 (0.104)

Kum LL (*α*, *β*, *γ*, *δ*)	*α* = 2.319 *β* = 5.749 *γ* = 2.182 *δ* = 7.903	0.201	1.071	0.161 (0.101)

Mo-LL (*α*, *β*, *γ*)	*α* = 6.064 *β* = 4.633 *γ* = 4.330	0.203	1.089	0.169 (0.109)

## Data Availability

The data used to support the findings of this study are included within the article.
